# Trichoscopy of Alopecia Areata: Hair Loss Feature Extraction and Computation Using Grid Line Selection and Eigenvalue

**DOI:** 10.1155/2020/6908018

**Published:** 2020-09-25

**Authors:** Sunyong Seo, Jinho Park

**Affiliations:** ^1^Department of Media, Graduate School of Soongsil University, 369 Sangdo-ro, Dongjak-gu, Republic of Korea; ^2^Global School of Media, Soongsil University, 369 Sangdo-ro, Dongjak-gu, Republic of Korea

## Abstract

Recently, the hair loss population, alopecia areata patients, is increasing due to various unconfirmed reasons such as environmental pollution and irregular eating habits. In this paper, we introduce an algorithm for preventing hair loss and scalp self-diagnosis by extracting HLF (hair loss feature) based on the scalp image using a microscope that can be mounted on a smart device. We extract the HLF by combining a scalp image taken from the microscope using grid line selection and eigenvalue. First, we preprocess the photographed scalp images using image processing to adjust the contrast of microscopy input and minimize the light reflection. Second, HLF is extracted through each distinct algorithm to determine the progress degree of hair loss based on the preprocessed scalp image. We define HLF as the number of hair, hair follicles, and thickness of hair that integrate broken hairs, short vellus hairs, and tapering hairs.

## 1. Introduction

### 1.1. Trichoscopy of Alopecia Areata

In recent, the hair loss population, alopecia areata patients, is distributed throughout the world and has a desire for treatments and diagnosis as hair loss progresses [1]. Hair loss affects the patient's confidence and morale and requires research to prevent and treat hair loss as quickly as possible [2]. To recover from alopecia areata, Minoxidil and Propecia are used to promote hair growth for men, but these methods are not the preferred treatment for patients with relatively low progression of hair loss due to the presence of unknown long-term effects and potential side effects [3]. Historically recorded images with a microscope provide a utility diagnostic method for measuring early FPHL (Female Pattern Hair Loss) [4].

One of the ways to treat hair loss, the scalp diagnostic method, can define and categorize the progress degree of alopecia areata and its indicators. Trichoscopy is a quick, noninvasive, cost-effective, bedside technique that provides key physical diagnostic information to assist in the accurate diagnosis of alopecia areata [5, 6]. In this paper, a scalp diagnostic method is performed based on the microscope image. In the image preprocessing section of the HLF extracting algorithm, we use the methods of image processing as statistical methods, complete automation, and semiautomation defined by Bonnet [7]. The aim of this research is to predict the condition of alopecia areata by extracting HLF from scalp images and measuring their scalp condition for those who are not subject to alopecia areata. In other words, the main purpose is to create objective indicators that allow nonpatients to determine their alopecia areata status through a microscope image.

In this paper, we introduce an algorithm for preventing hair loss and scalp self-diagnosis by extracting HLF (hair loss feature) based on the scalp image using a microscope that can be mounted on a smart device. The smart healthcare using wearable devices is making an outstanding growth together as these problems coexist. This industrial development has enabled health self-diagnosis throughout one's lives through the dissemination and high end of the smartphone. We have adopted a USB-connectable microscope and smartphone to provide simply distinguishable self-diagnosis solutions that can be served anywhere without space and time constraints for the public who are not familiar with medical knowledge.

### 1.2. Related Works

Researches continue to work on the detection and classification of certain diseases, including alopecia areata, using a microscope. Pollak et al. [8] conducted research to diagnose malaria through image recognition and machine learning algorithms. These automated image processing schemes have the advantages of standard definition, rapid diagnostic speed, expanded scanning area, and consistency for the diagnosis of a certain disease. Within the microscope, there are elements defined that affect alopecia areata such as vellus, terminal, microexclamation mark-type, monilethrix, and Netherton types. The state of hair follicles can be classified as a black dot, red dot, white dot, and yellow dot, and hair condition can be classified as broken hairs, short vellus hairs, and tapering hairs [9–11].

Trichoscopy has been used in advanced medical field to accurately diagnose the patient's scalp condition. Kim et al. [12] researched the evaluation of hair and scalp condition based on microscopy images analysis using a PCA [13] second principal component. Fang et al. [14] proposed Monte-Carlo simulation to estimate hair condition by changes and scales of hair condition in Chinese hair follicle state. This medical knowledge, however, tends to be inaccessible for the public to comprehend intuitively, which is valid for professionals, practitioners, or those with a certain level of background. Recent researches have shown to be a trend in image processing or machine learning-based hair segmentation [15], not to hair images taken with a microscope. These are based on an embedded system or GPU-enabled hardware, which is unapproachable for individuals to use them manually. Rolf [16] researched device and process called TrichoScan that estimates the number of hair, hair thickness, and hair density on the image and classify the anagen, telogen, vellus hair, and terminal hair. This research has preliminaries of cutting off target area and dyeing for the improved performance, which makes it more inaccessible, cumbersome, and time spending on the self-diagnosis system and is more likely to fail in the image with too many air bubbles or outside-crossing hair.

To solve these problems, we take a scalp image from a microscope and perform GLS (grid line selection) and eigenvalue computation based on computer vision that is runnable even on low-end devices. In this paper, we extract the HLF by combining a scalp image taken from the microscope using grid line selection and eigenvalue. First, we preprocess the photographed scalp images using image processing that adjusts the contrast of microscopy input and minimize the light reflection. Second, HLF is extracted through each distinct algorithm to determine the progress degree of hair loss based on the preprocessed scalp image. We define HLF as the number of hair, hair follicles, and thickness of hair that integrate broken hairs, short vellus hairs, and tapering hairs [17, 18]. Here, we define the hair follicle as an opened follicle with the hair. Although detecting yellow dot is one of the indicators of hair loss, we set the priority of counting the number of hair follicles as it also affects hair loss on how many hairs can grow in one follicle.

## 2. Methods

The input image taken with the microscope, top left in Figure 1, may have several noises in feature such as red dot, dyeing hair, and skin inflammation. The optimum preprocessing is carried out in order to minimize the distribution of these noises. After preprocessing, the algorithm is performed to extract the HLF. The preprocessing also enters separated inputs as the algorithm method to extract the features of each HLF is different.

Most of the scalp image does not look all intelligibly by the reflected light of the hair. In addition, there are cases where the hair crosses over each other or the hair in front covers the other hair; it is not recognized as itself. To cut out these problems, the image preprocess appropriate for each algorithm method is carried out as shown in Figure 1. The primary purpose of this research is to actualize a method of measuring the scalp of anyone's own by mounting a USB microscope to portable devices, such as smart wristband or smartphone, and adjust technologies that minimize the amount of computing for each preprocessing and algorithm methods.

### 2.1. Image Preprocessing

Input image that can be obtained from the microscope is defined as with a minimum HD ratio of 4 : 3, and we resize this input image to square size of 512. It is a common procedure to maintain the ratio in general to filter images when scaling is performed in the calculation of image processing before sampling according to the characteristics of downsampling or upsampling [19]. However, we had to resize to square size as the issue exists in eigenvalue computation, which will be described later. Then, the input image with RGB value was converted to greyscale, where the weight of *R* value was lowered relative to other values.

A morphologically reshaped image still has a black area shaded by a microscope and a hole in the hair that is reflected by the gloss of hair. Contrast stretching [20] is performed to solve these problems. The left-side picture of Figure 2 shows that the values of pixels corresponding to the full images are relatively centralized rather than the right-side picture. This means that it is evenly distributed regardless of the overall contrast of the image. The noises from this consequence should be distinguished between the feature and other nonfeature components and may alleviate some activities in defining the threshold parameter for binarization [21].

It can be seen that the values of adjacent pixels in the right picture of Figure 2 are biased to one side compared to the left picture after the contrast stretching. This confirms that the certain pixel values are recognized as inessential noise and shifted to adjacent pixel values and can smoothen the curve of the graph using a Gaussian filter [22]. In the case of graph converted to a gentle slope, as shown in Figure 3, it is more easygoing to find the optimum threshold parameter for binarization on a microscopy image.

HLF has its own algorithm to extract each feature. In order to extract hair thickness and the number of hair follicles, the hole in the hair reflected by gloss of hair and directional light of the microscope must be removed. Morphological Erosion [23] that is used for image denoising like salt and pepper makes more perfection by dilating the nonnoise and hair feature in an image. We could apply the methods as the holes in the image are classified as noise for adjacent pixel values. However, because Morphological Erosion would dilate even to the adjacent hair, so there are cases where multiple hairs are classified as one, so the preprocessing was not performed in the GLS Algorithm, which measures the number of hairs.

Up to this process, we constitute the definite boundary between the hair and scalp and the light reflected off the hair. Finally, all noise other than hair should be wiped out through image binarization, since only hair is comprehended as a feature in the image. Although we attempted to use the commonly applying adaptive threshold methods, we did segment the hair and other feature using the basic threshold as the black shaded area on the scalp is also recognized as a feature. The pixel value corresponding to the hair feature is separated to true and the remaining values in the image are false.

### 2.2. HLF Computation

The preprocessed image minimized the relationship between hair features and scalp and light reflected on the hair. The input value used to calculate HLF is the preprocessed image for each of the algorithm methods.

#### 2.2.1. Grid Line Selection for Hair Detection

The number of hair means countable hair in the image that can be seen with the naked eye, including broken hair, tapering hair, and normal hair. In this paper, only the hair that has been preprocessed in previous step is a unique feature with a value. For this hair feature, it is accomplishable to apply a Hough transform [24] ordinarily used in investigating the number of straight lines. We proceed with the skeletonization [25] that leaves only the center axis from each counted hair before applying Hough transform.

Hough transform has parameters whether the Hough space recognizes more *n* intersections as straight lines for each point of intersection area. Not only is it hard to find out the optimal parameters for transformation and detection, but also most of the hair is not straight out, curved, and waved; the number of hairs that have been detected were not properly computed. As shown in Figure 4(a), it can be confirmed through experiments that only 11 hairs have been detected by the Hough transform for line detection algorithm.

We used histogram-based methodology to detect the number of hair *h*. First, we arrange the *n* grid horizontally and vertically in the image. Next, extract all true values which are present and overpass on the gridline. Obtain the number of all true values from the *n* Grid defined as the following equation:

(1) $$\begin{array}{c} h=\frac{2\sum_{x\in B,B^{T}}\sum_{j=0}^{w}x_{j}}{n_{\text{grid}}+1}, \end{array}$$

where *B* = {*l*_1_, *l*_2_, *l*_3_, ⋯, *l*_*n*_}.

(2) $$\begin{array}{c} x_{j}=\left\{\begin{array}{c} 1,\;\text{if }x_{j}==\text{true},\\ \;0,\;\text{if }x_{j}==\text{false}. \end{array}\right. \end{array}$$

*n*_grid_ is a parameter that determines the number of grids, *B* is a set of index lines coinciding with *w*/*n*_grid_ in Figure 5, and *w* is the length of one side in the square image. The constant value of 2 is the ratio of an average length of all hair in the entire images, and it is assumed that about half of the length is constituted in this experiment. Equation (1) allows the number of hairs to be measured from the feature image. However, if the *x*_*j*_ and *x*_*j*+1_ values adjacent to the gridline are continuous in Equation (2), the calculation is fulfilled by treating them as one true value.

#### 2.2.2. Hair Follicle Detection

We proceed with the skeletonization of the preprocessed image. Skeletonized image in Figure 6(a) is a group of points with only one pixel thick on each line for *n* hair, the same as the method conducted in the Hough transform. For each skeletal hair, we extract pixels estimated as endpoints. Endpoints are specified as the points where the number of 8 neighbors is only 1 for skeletal hair and finally given the edge point of the image like Figure 6(b).

After the masking process, images are cropped to a certain size based on the endpoints presumed to be hair follicles, and the number of hair overpassing the edge of the cropped images could be estimated by each hair follicle. In this case, however, as the hair rooted in the hair follicles or is completely obscured so the hair follicle itself is ambiguous to recognize, it can be seen as a low performance through experiments.

The edge-based methodology is having difficulty in determining the crop size for an image, and the resulting performance in not respectable, so we used a clustering scheme. Clustering goes through the process using the *K*-means [26] algorithm based on the masked pixels. The input masked image was standardized to [0, 1] based on the resized size 512. We specified centroid *c*, which is the starting point for *K*-means, Gaussian distribution for the *x*- and y-axes, respectively.

(3) $$\begin{array}{c} \underset{S_{i}\in U}{\text{argmin}}\;\overset{k}{\underset{j=1}{\sum }}\underset{x\in S_{ij}}{\sum }{\left\|x-\mu_{ij}\right\|}^{2}, \end{array}$$

where *U* = {*S*_1_, *S*_2_, *S*_3_, ⋯, *S*_*n*_}, *S*_*i*_ = {*S*_*i*1_, *S*_*i*2_, *S*_*i*3_, ⋯, *S*_*ik*_}.

For the commonly used *K*-means, there is a problem that must first be allocated *k*, the number of start centroid, and the algorithm is processed. This could be resolved by compounding a hyper set *U* and loss function for the optimal set *S* to be obtained. First, we assumed that the number of all cluster sets to be calculated is *n*. For each cluster *S*_*i*_ belonging to *U*, we have the number of centroids from 1 to *n*. The sum of the Euclidean distances used to form the cluster with the optimal set *S*_*i*_ shown in Equation (3) is defined as the loss function. The cluster set with the least loss function is considered to be the optimum cluster set. The least loss function could be interpreted as the cluster set being constructed relatively speedily, and less Euclidean distance calculated in all cases constituting the cluster is small, on average. All data *x* must belong to the *S*_*i*_ set, where cluster *S*_*i*_ can be a null set. *μ*_*ij*_ is the centroid of each cluster *S*_*i*_. The number of clusters that are not the null set of the *i*-th cluster set with the least loss function is finally determined as the number of hair follicles as shown in Figure 6(c).

#### 2.2.3. Hair Thickness Computation

First of all, we compute the number of true values from the preprocessed image. And we estimate the *n* contoured image through contour detection [27] from the image with only the hair remaining. And we calculate the eigenvalue [28] and the amount of green line length in Figure 7, for each *i*-th contoured image. The calculated eigenvalue is an indicator of the percentage of proportion in the image represented by one hair. If the width and height of the input were different, the eigenvalue of the hair would have been different depending on the stretched length of the horizontal and vertical, respectively, which is why the resizing was carried out as a square in the preprocessing step. The hair thickness *t* can be approximated by averaging each eigenvalue in the cropped image and excluding the expanded amount of true values generated in the Morphological Erosion.

(4) $$\begin{array}{c} \Lambda \left(p\right)=1+\ln\left(1-\frac{\bar{\lambda_{p}}-1}{e}\right), \end{array}$$

(5) $$\begin{array}{c} E\left(p\right)=\Lambda_{p}\cdot h\cdot \frac{s}{c}, \end{array}$$

(6) $$\begin{array}{c} t=\alpha \left(\frac{\text{area}}{h}-E\left(p\right)\right). \end{array}$$

$\bar{\lambda_{p}}$ is the average of the eigenvalue pulled up through contour detection for each *n*-th image in Equation (4). $\bar{\lambda_{p}}$ is standardized to [0, 1], which defines the hyperparameter values divided by denominator *p*. In Equation (5), *h* is the number of hairs estimated by GLS and indicates the extent to which the dilated area affected hair. *c* is the number of all contours detected in the contour detection algorithm, and *s* is the value that scales the approximate number of pixels in practice dilated by Morphological Erosion in the image. We initialized *s* as (erosion size)∗(length of one side of resized image∗2) used in the parameter of the erosion algorithm. Area is the number of true values; that is, how many hair features exist in the image in Equation (6). *α* is a constant that converts the values into micrometers. Finally, the *t* can be inferred from the scalp images through Equation (6).

## 3. Evaluations and Results

Evaluation proceeds based on the microscopy image taken directly from the Galaxy Tab S4. The microscope can be magnified from 20x to 800x. We used two types of microscope for evaluation. Both microscopes preserve the same scale on measuring but yield the discrete color pixel values, being more reddish than the other one. The evaluation indicators are defined of the number of hair, hair thickness, and hair follicles, respectively. Of the scalp images, including from 20s to 40s of men and women, one hundred test sets are randomly treated for evaluation.

In this paper, the algorithm is evaluated by the accuracy of HLF for a single shot image rather than measuring precision and recall for each hair. The accuracy of the number of hair and hair follicles are measured based on the truth label appraised directly by the naked eye. Hair thickness is measured manually using a hand-made hair thickness measurement tool. The number of hair truth is measured which is not too disturbed by noise on the naked eye, overpassing the image including itself. Hair follicles are measured in the number of itself with a hair except in the case of hair follicles such as red dots, black dots, and yellow dots that inflame the hair from growing. We also measured follicles that exist on the edge of the image almost seen faintly.

In defining truth values in the evaluation indicator, the variances of truth values are shown to be significantly spacious depending on the measurer, especially for the number of hair follicles. This is because if several hair follicles appear to be overlapped as one, or if hair passes through the hair follicles, so it is unable to visually discriminate with the naked eye; various opinions were reflected in each different measurer. It was also found that the error occurred because the presence of hair follicles at the edge of the image was extremely, subjectively judged.

Keep in mind that the column input data in Table 1 is the same as the input name of Figure 8. As shown in Input (b) in Figure 8, hair follicles are difficult to measure when hair that overpasses an image is obscuring the hair follicles exactly at a certain point. Input (d) in Figure 8 shows that there is an outstanding error in measuring the number of hair that are out of focus as it blurred a significant portion of the images, causing a lot of noise, also in the case of hair dense on the left difficult to distinguish with the naked eye. However, the average of the whole data with a various test data is performed excellent accuracy of 96.51%. In contrast to the whole data, the case of error rate of each data in hair follicles recorded a comparatively low figure of 84.07% and 82.33%, which can be shown in Figure 9. This result is considered to be a consequence where deviation is vast for each data. Within a dataset, the maximum error of the number of hair is 16 and follicle is 4, interpreting that errors are quite extensive for some noisy images.

Of the data in Figure 10, input (a) is stably taken, and in the case of input (b), it is taken with the microscope shaken or out of focus, resulting in superfluous blur and noise. Even though the preprocessing was performed as the noise is too high, we could not accurately leave the hair as a feature, and as a result, we could find out through the experiment that the value of the hair stands out significantly when we carried out the algorithm. In the case of input (c), it can be seen that there is plenty of broken hair in the image by artificially cutting off short. Remarkably, the number of hair follicles and hair thickness are decently measured in this case; only the error appears in measuring the number of hair. On input (d), hair that does not have hair follicles is intersected to hinder hair follicles, and the focus is out of hair on desire, resulting in noise. On the contrary, the number of hair is measured and improved than relatively noisy input (b), in which it is confirmed that there is an error with the number of hair follicles and hair thickness.

The algorithm computing time for the whole process showed the performance of approximately 0.2 seconds per image in the Ryzen 5 2600 environment, including loading time. When dispatching between smartphones and PCs, the response time on client was less than 2 seconds. In the practical application level, we compare the back hair of the head, which is a healthy portion of the whole head, and an alopecia target portion to calculate the relative figure of own head.

## 4. Conclusion and Future

It is important that hair loss caused by both congenital and acquired factors be recognized by the patient themselves and with appropriate diagnosis be given a nonexcessive treatment, such as drug overdose, for its progress. In an acquired point of view, hair loss is influenced by diet, surrounding environment, psychological state, etc. which varies in progress depending on gender [29–32]. We automatically estimate the feature from a large amount of scalp images by extracting HLF using only one singular microscopy image. Also, by recording a historical HLF identified as a result of hair loss, the cause of alopecia areata can be analyzed through time series analysis [33], granger causality [34], ARIMA [35], or artificial intelligence.

We enabled a novel diagnosis of alopecia areata by combining computer vision and image processing to extract HLF using a microscopy image that can be worn on a smartphone through this paper. This, as shown in the evaluation section, has enabled highly distributed public indicators with large variance as a consistent evaluation indicator through the algorithm and also allow the patient's scalp condition to be stored along the timeline by historically measuring the feature of the scalp. It would derive a new correlation between alopecia areata and scalp condition as there is no specific sign or condition for judging hair loss progress. By providing HLF results to the patients, this research let them follow up and be consciousness of handling the hair loss progress.

Computer vision studies use various fields in vision machine learning studies for extracting specific features, variables, parameters, and object detection from the image. Of course, the accuracy of computer vision AI based on machine learning shows high performance when using a fully prepared dataset and validated model, but convolutional neural network-based AI still requires a tremendous amount of parameters [36]. To address this, researches continue to be conducted that record high accuracy with minimal AI model sizes [37], but to date, it is assumed that it still has an issue on fitting into solutions or light portable devices. In addition, in order to create a model with exceptional performance in a particular field, the engineer needs a large amount of dataset for a preprocessed image, which enables us to create an image with the feature as an input dataset through this paper. Our following research aims to build artificial intelligence that can extract more types of HLF with an only microscope image, being not attached to any specific sensors.

## Figures and Tables

**Figure 1:** Algorithm pipeline. Top left: input scalp image that is taken from a microscope. Blue block: image preprocessing. Orange block: key method for HLF extraction.

**Figure 2:** Contrast stretching comparison.

**Figure 3:** (a) Filtered and (b) contrast stretched filtered.

**Figure 4:** Hough transform: (a) result of line detection and (b) Hough space.

**Figure 5:** Visualization of GLS.

**Figure 6:** Follicle detection algorithm.

**Figure 7:** PCA algorithm visualization. Green line: eigenvector with the largest eigenvalue used in this method. Eigenvalue expands as the hair reaches out on the image. Blue line: second eigenvector in PCA which has a vertical direction of the primary eigenvector.

**Figure 8:** Process from preprocessing to the HLF extraction algorithm. Input (a): evaluated with a good performance in hair follicle detection. Input (b): evaluated with a low performance in hair follicle detection. As the hair overpasses the other hair in skeletal stage, the hair features disappeared or overlapped, so the algorithm is not properly performed through the input of the preprocessing image. Input (c): evaluated with a good performance in the number of hair with different types of microscope. Input (d): evaluated with a low performance in the number of hair. The image seems like to have out-focused noise to a blurred hair. Input (e): evaluated with a good performance in estimating hair thickness. Input (f): evaluated with a low performance in estimating hair thickness. The contour detection does not perform properly on Input (f), which makes an eigenvalue to incorrect value.

**Figure 9:** Prediction result figure of test dataset.

**Figure 10:** Various test images.

**Table 1:** Evaluation of Input data in Figure 8. Bold data are assumed as bad experiment results and italic data as good experiment results.

	Input (a)	Input (b)	Input (c)	Input (d)	Input (e)	Input (f)	Dataset
Hair truth	18	20	23	23	17	25	19.59 (avg)
Hair prediction	15.42	22.49	22.73	12.97	15.21	23.12	19.04 (avg)
Hair difference	2.59	2.49	*0.27*	**10.03**	1.79	1.88	*3.13*
Follicle truth	9	8	7	7	8	7	8.15 (avg)
Follicle prediction	9	12	8	7	10	6	8.49 (avg)
Follicle difference	*0*	**4**	1	*0*	2	1	*1.44*
Thickness truth	53.8168	67.0311	72.8527	76.7309	66.6854	60.6011	—
Thickness prediction	61.0024	65.3314	67.3158	87.0331	58.4213	60.4601	61.98
Thickness difference	7.1856	*1.6997*	5.5369	**10.3022**	**8.2641**	*0.141*	—
Total accuracy	*90.75*	78.34	*92.31*	**80.99**	84.03	*92.65*	*96.51 (avg)*
							*83.20 (diff)*

## Data Availability

The data used to support the findings of this study is available from the corresponding author on reasonable request.
